The article "Blockchain-Based Optimization Model for Evaluating Psychological Mental Disease and Mental Fitness" was published in 2022. Journal: Comput Intell Neurosci.

# Blockchain-Based Optimization Model for Evaluating Psychological Mental Disease and Mental Fitness

**DOI:** 10.1155/2022/8657313

**Published:** 2022-07-14

**Authors:** Jayashree Rajesh Prasad, Shashikant V. Athawale, Roshani Raut, Sonali Patil, Sheetal U. Bhandari, Mohd Asif Shah

**Affiliations:** ^1^School of Engineering, MIT Art, Design and Technology University, Pune 412201, Maharashtra, India; ^2^Department of Computer Engineering, AISSMS COE, Savitribai Phule Pune University, Pune, India; ^3^Department of Information Technology, Pimpri Chinchwad College of Engineering, Akurdi, Savitribai Phule Pune University, Pune, Maharashtra, India; ^4^Department of E & T/C Engineering, Pimpri Chinchwad College of Engineering, Pune, India; ^5^Kebri Dehar University, Somali, Ethiopia

## Abstract

The current work describes a blockchain-based optimization approach that mimics the psychological mental illness evaluation procedure and evaluates mental fitness. Combining lightweight models with blockchains can give a variety of benefits in the healthcare business. This study aims to offer an improved review and learning optimization technique (SPLBO) based on the social psychology theory to overcome the biogeography-based optimization (BBO) algorithm's shortcomings of low optimization accuracy and instability. It also creates high-accuracy solutions in recognized domains quickly. To retain student individuality, students can be divided into two groups: Human psychological variables are incorporated in the algorithm's improvement: in the “teaching” step of the original BBO algorithm; the “expectation effect” theory of social psychology is combined: “field-independent” and “field-dependent” cognitive styles. As a consequence, low-weight deep neural networks have been designed in such a manner that they require fewer resources for optimal design while also improving quality. A responsive student update component is also introduced to duplicate the effect of the environment on students' learning efficiency, increase the method's global search capabilities, and avoid the problem of falling into a local optimum in the first repetition.

## 1. Introduction

Machine learning algorithms can effectively identify possible features from the provided data; therefore, they do not require any hand-crafted characteristics throughout the simulation. Neural network models can effectively identify possible features from the provided data; therefore, they do not need any manual features throughout the prediction phase. Teaching-learning-based optimization (TLBO) is a new heuristic algorithm proposed by author [1]. The algorithm simulates the teaching and learning process design of teachers and students. Students can acquire knowledge from teachers' teaching and understanding through interaction between students. The TLBO algorithm has the advantages of few parameters, simple structure, and fast solution speed, and its competitiveness mainly comes from the ingenious design of the teaching and learning stages. Compared with other typically improved intelligent optimization methods, the TLBO algorithm also shows its outstanding performance and advantages. However, simultaneously, it holds a large number of drawbacks such as to take up a lot of resources like storage and memory. It is a time-consuming procedure because it requires several iterations and thus processing takes a longer time than usual, which are the main concerns of the TLBO algorithm. Furthermore, as compared with the Genetic Algorithm (GA), TLBO allows the population to learn from the optimal individual in the teaching phase, thereby improving the convergence speed of the algorithm; compared with Particle swarm optimization (PSO), for a single operator, TLBO introduces one more learning stage than PSO, which is beneficial to improve the exploration ability of the algorithm; compared with Cuckoo Search (CS), TLBO provides interactive learning in the learning stage method [2, 3]. It is precisely because TLBO has these advantages that scholars have never stopped studying it since the algorithm was proposed. However, the TLBO algorithm also has shortcomings such as low optimization accuracy, poor stability, and slow convergence speed. Many scholars have improved it from multiple perspectives. The improvement direction is mainly divided into three aspects: improving the teaching process, introducing weights or adaptation factors, and combining with other intelligent optimization algorithms. Among them, the improvement of the teaching process refers to adding a self-study stage or introducing new learning rules based on the original teaching stage and learning stage [4]. Collaborative Learning Model (CLM) is used for the learning phase. In the CLM method, to guide the learners effectively, the teacher will adaptively update its position according to the neighborhood information in the self-learning stage [5]. A novel optimization algorithm based on autonomous learning was proposed and the authors remodeled the proposed algorithm according to the three stages of the teaching process: teacher's learning, mutual learning, and self-learning between students. The literature introduced a teaching and learning algorithm with logarithmic helical strategy and triangular mutation rule (LNTLBO) to enhance the exploration and development ability in the learning stage [6]. The literature proposed a teaching and learning optimization algorithm based on multi-reverse learning, established a hybrid reverse learning model, and added a self-learning stage based on search boundary guidance, making the algorithm more robust to global search and local detection capability [7].

The literature adopted a different feedback learning stage to speed up the convergence, further recording the previous generation teachers and communicating with the current teachers to provide comprehensive feedback to the learners and supervise the learning direction to avoid wasting previous generation computation quantity [8]. The literature let teachers perform dynamic random search algorithms in the later stage of the algorithm to improve the ability of the optimal individual to explore new solutions [9]. For improvements in introducing weights or unknown parameters, the literature has proposed Advanced Teaching Learning-Based Optimization (ATLBO). New weight parameters were introduced to improve the accuracy and speed up convergence [10]. Authors have proposed the nonlinear inertia-weighted teaching-based optimization algorithm (NIWTLBO) [11]. The algorithm introduces a nonlinear inertia weighting factor into the basic TLBO to control the learner's memory rate. It uses a dynamic inertia weighting factor to replace the original random number in the teaching and learning stages. The literature introduced the crossover operator of the difference algorithm in the “teaching” stage and the “learning” stage, and at the same time carried out an adaptive local search according to the normal distribution around the elite individuals to improve the convergence speed and solution accuracy of the algorithm [12]. To enhance the performance of TLBO, many scholars try to integrate it with other optimization algorithms. The literature added an error correction strategy and Cauchy distribution (ECTLBO) in TLBO, where Cauchy distribution is used to expand the search space and correct wrong to avoid detours for a more accurate solution [13]. The literature combined harmony search with the teaching and learning optimization algorithm and proposed a hybrid optimization algorithm (HHSTL) based on harmony search and teaching and learning optimization, which enabled the algorithm to solve more complex problems [14]. The literature proposed an improved teaching and learning optimization algorithm (ITLBOBSO) incorporating the idea of brainstorming and introduced Cauchy mutation and a random parameter associated with the number of iterations in the operator to improve the performance of the algorithm [15]. The literature proposed a hybrid search algorithm named HSTLBO, in which HS mainly aims to explore unknown regions. In contrast, TLBO aims to rapidly develop high-accuracy solutions in known areas [16].

TLBO is a new heuristic algorithm that takes people as the main body of activities and simulates teaching phenomena. The improvement of TLBO mainly focuses on manufacturing the teaching process and combining it with other algorithms. However, very little consideration is given to people's psychological and emotional factors, such as considering the influence of psychological factors on behavior results from the perspective of people; individuals with different personalities show different states in the same environment. This improvement makes the algorithm have a specific revision in the optimization performance, but there is still room for improvement in stability and convergence speed.  Figure 1 shows the mental state relation with the students.

To further improve the algorithm's performance, this paper focuses on social psychology, considers human emotions and behaviors, and simulates the impact of human psychological factors on the results in the teaching process. We apply the social psychological theory to algorithm improvement. First, the “expectation effect” theory is added to the teaching stage [17]. The theory states that in interpersonal interactions, one party has expectations of the other party. The party that has expectations will treat the other party as he expects, thereby causing changes in the other party's behavior. It is reflected in the algorithm that the individual teacher provides one-to-one teaching to the students with good fitness value, and the teacher guides the students who are taught one-to-one. They also change their learning behavior and begin to learn from other students. The theory of “field independence-field dependence” is added [18]. This theory divides people's cognitive styles into “field-independent” and “field-dependent” according to their different degrees of dependence on the external environment. Starting from the actual situation, considering the different cognitive styles of international students, we simulated field-independent and field-dependent students and adopted different learning strategies. After being taught by teachers and learning from each other, students need to digest knowledge points and evaluate their rankings. The learning method is extended or adjusted according to the ranking situation, and thus the self-learning method adjustment phase is added after the learning phase [19]. Bandura's “self-regulation theory” exists in psychology, which shows that self-regulation includes three processes: self-observation, self-judgment, and self-reaction. According to this theoretical score, different self-regulation strategies are used for students in various positions to achieve a better state. Finally, a series of test functions prove that the improved algorithm has obtained better performance in terms of optimization accuracy and convergence speed. The TLBO method has a number of flaws, including poor optimization accuracy, instability, and slow convergence time. It has been improved by a number of academics from a number of views.

Adding social psychology to algorithm improvement also has specific innovations in intelligent optimization algorithm improvement. The current work describes a blockchain-based optimization approach that mimics the psychological mental illness evaluation procedure and evaluates mental fitness. Combining lightweight models with blockchains can give a variety of benefits in the healthcare business. This study aims to offer an improved review and learning optimization technique (SPLBO) based on the social psychology theory to overcome the biogeography-based optimization (BBO) algorithm's shortcomings of low optimization accuracy and instability. Since people are a complex system affected by their psychological state, they will take timely measures to adjust their behavior to seek a sense of self-protection. Therefore, compared with the improved methods of other intelligent optimization algorithms, incorporating human psychological factors can make the algorithm improvement more flexible and allow the algorithm to balance global search and local search. This research paper, focusing on the defects of low optimization precision and slow convergence speed when solving complex optimization problems of the teaching and learning optimization algorithm, from the perspective of social psychology, combined with the changes of people's psychological emotions, improves the original teaching and learning optimization algorithm.

## 2. Blockchain-Based Teaching and Learning Optimization Algorithm (B-TLBO)

B-TLBO is an algorithm designed to simulate the two stages of teacher teaching and student learning in the process of simulating class teaching. It uses the entire population as a class, the best individuals in the population as teachers, and the other individuals as students. The concept of the B-TLBO algorithm comes from the replicated class's teaching process; to better replicate the new state of middle school students in the teaching phase, an adaptable student updating factor is incorporated, and the method is expected to produce superior results. The algorithm is divided into the “teaching stage” and the “learning stage.”

Figure 2 depicts the B-TLBO method that relies on the teaching process of a repeated class and has two stages as discussed. The “teaching stage” refers to when the entire student body learns from the teacher, while the “learning stage” corresponds to when the students learn from one another. The total level of the population is improved by the co-evolution of these two stages. In this study, *N* denotes the total number of students (i.e., the population size), and *d* is the number of subjects studied by each student (i.e., the individual dimension). Each student is identified as *S*_*i*_ = {*S*_1_, *S*_2_, *S*_3_, *S*_*n*_} with the fitness function *f* (*x*_*i*_) indicating the student's grade; the higher the fitness value, the higher the grade. The specific content of the algorithm is described in two stages, namely the teaching stage and the learning stage, respectively. The best fitness value for each of the iteration has been selected to convey the knowledge to the students in the best possible way; similarly, the learning stage is the technique of combined learning of all students in a group after the accomplishment of the teaching stage and here the fitness function is chosen to select the best student among the students. Hence, we can complement that the two methods in the BTLBO algorithm are employed for the enhancement of the fitness functions. The two techniques are listed as follows:

### 2.1. Teaching Phase

In the teaching phase, the individual with the best fitness value for each of the iteration will be selected as the teacher *T*_*X*_. The teacher imparts knowledge to the students to improve the average grade of the whole class. He hopes that the overall middle position of the class *T*_*M*_ is close to its *T*_*X*_. Therefore, the teaching method design is given by formula (1):

(1) $$\begin{array}{c} t_{i,\text{new}}=t_{i}+r_{i}\left(t_{x}-t_{f}t_{m}\right), \end{array}$$

where *t*_*i*,new_ represents the new state of student *i* after learning in the teaching stage; *t*_*i*_ is the original state of student *i* before learning; *r*_*i*_ is a random number on [0, 1]; the influence degree of the value generally takes 1 or 2. After the teaching phase is completed, the students update the knowledge reserve, and each student decides whether to update according to the new state or the original state. Take the minimization problem as an example:

(2) $$\begin{array}{c} \text{if }f\left(t_{i,\text{new}}\right)<f\left(t_{i}\right). \end{array}$$

### 2.2. Learning Stage

This stage simulates the process of mutual learning among students after the class is over. To further improve their learning level, students communicate with other individuals in the class. Student_*i*_ randomly selects student_*j*_, compares the fitness values of the two students, and subtracts the second-best student from the position of the best student. Taking the minimum optimization problem as an example, the learning is carried out in the following way:

(3) $$\begin{array}{c} t_{i,\text{new}}=\left\{\begin{array}{c} t_{i}+\text{rand}\left(t_{i}-t_{j}\right),\\ f\left(t_{i}\right)<f\left(t_{j}\right),\\ t_{i}+{\text{rand}}_{i}\left(t_{j}-t_{i}\right), \end{array}\right) \end{array}$$

where rand_*i*_ is a random number on (0, 1). After the learning period is over, perform the same update operation on the students as in the teaching period again.

## 3. Teaching and Learning Algorithms Based on the Social Psychological Theory

To further improve the algorithm's performance, this paper improves three aspects of the teaching and learning algorithm from the perspective of human emotion and psychology, combined with the social psychology theory. Firstly, the “expectation effect” is introduced in the teaching stage, and students who bear different expectations will adopt different learning strategies. The idea of “field independence-field dependence” is presented at the learning stage to distinguish the differences in the learning styles of other students. Finally, considering the actual teaching situation, a self-learning method adjustment phase is added after the teaching and learning phases to adjust students' learning methods in time.

### 3.1. Introducing the “Expectation Effect” Theory to Improve the “Teaching Stage”

Teachers always have higher expectations for students with relatively good grades in daily teaching. To get better grades, teachers will take one-on-one teaching or set up advanced courses and other methods. An expectation is a judgment about oneself or others that one expects to achieve a specific goal or meet a confident behavioral expectation. Students with better grades will take active measures to study harder to live up to teachers' expectations after teachers have focused on them. For example, they can improve themselves by increasing their study time and sharing their learning experiences with their classmates. This phenomenon is known in social psychology as the “Pygmalion effect” or the “expectation effect.” An expectation is a judgment about oneself or others that one expects to achieve a specific goal or meet a confident behavioral expectation. The behavioral outcome that results from expectations is the expectation effect. In this statement, the author wants to express the psychological aspect about the person's expectation of the other individual, and it means that an expectation is a kind of judgment about a person or somebody that is referred as the “expectation effect.” Expectation emphasizes the activity process of the individual's psychological stimulation, while the expectation effect focuses on the behavioral results produced by psychological stimulation. The literature introduced this theory into business management practice [20]. The results show that managers' expectations of subordinates and how they treat associates determine the work performance and career progress of these subordinates to a large extent. Inspired by this, the algorithm is improved: Classify students whose grades are above the class average as outstanding students, and learn by combining one-to-one teaching with teachers and learning from other students, as shown in formula (4):

(4) $$\begin{array}{c} t_{i,\text{new}}=t_{i}+r_{i}\left(t_{x}-i_{x}\right)+r_{i}\left(t_{r1}-i_{r2}\right). \end{array}$$

Students whose grades are below the class average will study according to formula (5):

(5) $$\begin{array}{c} t_{i,\text{new}}=t_{i}+r_{i}\left(t_{x}-f_{t}*\text{mean}\right). \end{array}$$

Among them, *t*_*r*1_ and *t*_*r*2_ are the status of any two students in the class, and mean is the average level of the classmates. When the fitness value of a student is higher than the average, it will bear the high expectations of the teacher. It can be seen from formula (4) that to meet the teacher's expectations in the learning process, in addition to relying on its own knowledge state  *t*_*i*_, the student_*i*_ also adopts one-to-one learning from the teacher.

Compared with formula (1), the student refers to the average difference between the teacher and the class in the learning process. Under this learning method, the space for excellent students to improve their grades is limited, which will reduce the speed of the algorithm converging to the optimal solution. The strategy of one-to-one learning from teachers is added to the improved formula (4), which increases the influence of teachers on students. This design allows outstanding students to approach teachers quickly and enables students to jump out of their limitations. To solve the problem of poor local search ability of the algorithm and to speed up the algorithm's convergence, a strategy of learning from classmates is added to equation (4). Students with an average score or above exchange experience with any classmate in the class, which improves themselves and helps others, improve their performance, thereby narrowing the gap between classes and accelerating the process of convergence of the entire population to the optimal value. When student's fitness value is lower than average, he does not bear the teachers' high expectations, and so his learning style will not change.

### 3.2. Introduce the “Field-Independent-Field-Dependent” Theory to Improve the “Learning” Stage

The concept of “field independence-field dependency” is introduced throughout the learning stage to distinguish between students' learning styles. In the learning phase of the standard teaching and learning algorithm, individual students learn in a unified way. However, in reality, students with different personalities take different learning styles. For example, some students are introverted and more independent and tend to accumulate experience in learning alone; some are extroverted, good at socializing, and like to gain knowledge in discussing and communicating with others. These two types of students are called “field-independent” and “field-dependent” types in social psychology, respectively. The two concepts of field independence and field dependence originate from the research on perception in literature. Field-independent people tend to refer to themselves when judging objective things and are not easily influenced and interfered with by external factors; field-dependent people tend to refer to the outside to process information and are less independent and easily influenced by the outside world. Due to differences in cognitive styles in learning activities, field-independent and field-dependent students tend to have different learning strategies. The knowledge sources of field-independent students are mainly composed of their knowledge accumulation and discussions with very few classmates; the knowledge of field-dependent students primarily comes from a part of their knowledge and extensive social discussions. In terms of algorithm design, considering that different students are affected by the outside world at different levels, a 0-1 matrix *W*_*i*_ is randomly generated to simulate field-independent (1) and field-dependent (0) students and take other learning methods for them. Strategies: Field-independent students study with the learning strategy of formula (2); field-dependent students study according to the following strategy:

(6) $$\begin{array}{c} t_{i\text{,new}}=\left\{\begin{array}{c} f_{ti}<f_{tj}:f_{t}*t_{i}+r_{i}\left(t_{x}-i_{x}\right)+r_{i}\left(t_{r1}-i_{r2}\right),\\ f_{ti}>f_{tj}:f_{t}*t_{i}+r_{i}\left(i_{x}-t_{x}\right)+r_{i}\left(t_{r3}-i_{r4}\right). \end{array}\right) \end{array}$$

It can be seen from formula (6) that *j*-*X*, 3*r*_*X*_, and 4*r*_*X*_ are three randomly selected students, *r*_1*i* _ and *r*_2*i*_  are random numbers on [0, 1], and *t*_*f*_ is a scale factor, which is used to reduce self-esteem at the previous moment. The technique works best when the *f t *value is set to 0.3 after several iterations. When WI is 1, it means that the individual student in *X* is field-independent, and in the learning stage, it learns according to the learning method of the original algorithm and completely retains its own state at the previous moment. When the value of WI is 0, it means that the individual student *t*_*i*_ is field dependent. Field dependence-field independence is a form of learning control that has been examined. It refers to the degree to which humans are influenced by inner or environmental stimuli when organizing themselves in time and making precise discriminations of their surroundings. Individuals who are field reliable are better at learning social content and doing it in a social context. People who work in the field in an independent manner are less reliant on being given a system to follow and are more self-motivated. In addition to randomly selecting a student to study, it will also exchange experience with other students and absorb some other people's knowledge to improve their own performance. At this time, the student *t*_*i*_ only retains part of their own state. Compared with the middle school stage of the original algorithm, this design weakens the influence of the state at the previous moment, and at the same time enhances the communication between individuals, reduces the probability of the algorithm falling into the local optimum, and maintains the diversity of understanding. Since the other half of the particles completely retain their own state, the convergence speed of the algorithm is also guaranteed. To verify the impact of improving the learning stage on the diversity of students, the program breakpoints are set in the learning stage, and the running results are shown in Figure 3.

Select some test functions in Figure 3, draw the student position map when the algorithm iterates 30 times, and compare the improved algorithm with the original B-TLBO; we can find that the diversity of students has been greatly improved.

### 3.3. Join the Self-Learning Method Adjustment Stage

Students need to have a precise understanding of their learning situation after two stages of learning through teacher teaching and communication with students. Therefore, self-assessment and regulation play an indispensable role in efficient learning. Bandura proposed the theory of self-regulation in the social learning theory emphasizing the internal reinforcement process of the individual [21]. Self-regulation includes three primary functions: self-observation, self-judgment, and self-reaction. People observe self-behavior according to social activities' standards, judge the gap between self-behavior and standards, and make positive or negative evaluations of self based on self-assessment.

The individual will have various inner experiences, such as self-satisfaction, self-blame, and criticism, resulting in self-regulation. People can use the effects of self-regulation to adopt more appropriate strategies to achieve their goals. Based on this theory, this paper adds a self-learning method adjustment stage which means earning information or skills via one's personal endeavors rather than through official instruction; after the teaching and learning stages in self-learning, we acquire observation, judgment, and consciousness which are efficient for boosting ones morale. It also creates high accuracy solutions in recognized domains quickly, providing students with a platform for self-reflection and timely adjustment of learning strategies. The specific settings of the self-learning method adjustment stage are as follows: after the teaching stage and the learning stage, the average score of the overall students is calculated, the individuals whose scores are higher than the average score are classified as excellent individuals, and the average score of the beautiful students is calculated. The class is divided into three categories based on the overall average score and the average score of outstanding students:

When the student's grade is higher than the average score of the excellent students, the student is an excellent student, which proves that his learning method is efficient; thus, the student will continue to study with his own learning method, as shown in formula (7):

(7) $$\begin{array}{c} t_{i,\text{new}}=t_{i}. \end{array}$$

When a student's grade is lower than the average grade of outstanding students, but higher than the overall average grade of the class, the student is an ordinary student, which proves that his learning method is partially effective, but there is still room for improvement, and the learning method can be fine-tuned to obtain better grades, such as formula (8) shows:

(8) $$\begin{array}{c} t_{i,\text{new}}=t_{i}+\left(t_{i}^{\min}+t_{i}^{\max}\right)\left(t_{r1}-t_{r2}\right). \end{array}$$

Among them, *t*_*r*1_, *t*_*r*2_ are (0, 1) random numbers, and *t*_*i*_^min^ and *t*_*i*_^max^ are the upper and lower bounds of student *i*, respectively. When the student's grade is lower than the average score of the class, it proves that the learning method is ineffective, and the learning strategy needs to be changed to a great extent. Here, the reverse learning method is used, as shown in formula (9):

(9) $$\begin{array}{c} t_{i,\text{new}}=\left(t_{i}^{\min}+t_{i}^{\max}\right)-t_{i}. \end{array}$$

The self-learning method adjustment stage enables individuals to make full use of the population information and adopt a better strategy to update. *t*_*i*_^max^ and *t*_*i*_^min^ represent the sum of the upper and lower bounds of student *i*, which provides a greater possibility for student *i* to change. Therefore, a fine-tuning random number *t*_*r*1_ is added to equation (8), such that individuals can still maintain diversity while converging. In formula (9), the sum of the upper and lower bounds is used to subtract the value of the previous state of the individual, which completely changes the position of the individual, thereby increasing the efficiency of the algorithm optimization. Putting this process after the learning stage can help individuals discover their own deficiencies in time and make adjustments quickly. It reduces the probability of bad solutions appearing in the iterative process, which helps improve the optimization speed and accuracy of the algorithm. In addition, since the B-TLBO algorithm idea originates from the teaching process of the simulated class, to better simulate the new state of middle school students in the teaching stage, an adaptive student update factor is introduced to expect the algorithm to obtain better results.

## 4. Experimental Results and Analysis

In this part, the performance evaluation of the algorithm adopts the exact maximum fitness evaluation time to evaluate the optimization accuracy of the algorithm. The proposed theory may be used to enhance the teaching and learning methods in the early stages of learning, as well as to solve more sophisticated optimization issues such as dynamic vehicle route optimization, parameter optimization in numerous domains, and so on. For each test function, the SPB-TLBO, B-TLBO, PSO, GA, and IA algorithms are run independently 30 times to obtain the optimal solution, worst solution, mean, and standard deviation, respectively.

### 4.1. Datasets

These archives and repositories include datasets that may be used for research purposes. Read the terms of use carefully to verify that you are using the data according to the standards set out by the data originator or repository.

#### 4.1.1. Inter-University Consortium for Political and Social Research (ICPSR)

Data from social science research may be found in more than 500,000 digital files made available by ICPSR. Science, history, and gerontology are among the many disciplines represented. Other topics of interest include criminology, ageing, and healthcare issues in the public and in the military and foreign policy. Moreover, included are topics such as early childhood education and ethnic minorities in the United States of America. Please contact the Social Science Data Archive for help with ICPSR data.

#### 4.1.2. Data Archive on Substance Abuse and Mental Health

Documentation linked to the collection, analysis, and distribution of behavioral health data is provided by the Substance Abuse & Mental Health Data Archive (SAMHDA). Various data formats, including SAS, SPSS, State, and others, may be downloaded.

#### 4.1.3. Data Repository for Criminal Justice Research and Analysis

The preservation, upgrading, and sharing of computerized data resources; research based on archived data; as well as specific courses in quantitative analysis of criminal justice data are all part of the NACJD's objective to help researchers better understand the field of criminal justice.

#### 4.1.4. Odum Institute's Data Verse

Researchers may use the Odum Institute's data management, archiving, and preservation services. Machine-readable data accumulated over more than a century may be found at the Institute. Datasets may be browsed and searched.

Based on the above four datasets, we are going to see how well the method works in this paper. This paper looks at the standard accuracy rate (*P*), the recall rate (*R*), and the microaverage *F*1 as indicators of how well the model does; the formula for this is:

(10) $$\begin{array}{c} \text{Precision}\left(p\right)=\frac{\text{true Positive}}{\text{True Positive}+\text{false Postive}},\\ \text{Recall}\left(R\right)=\;\frac{\text{true Postive}}{\text{True positive}+\text{False negative}},\\ F1=\frac{2PR}{P+R}. \end{array}$$

In this paper, we evaluate four data on the entire evaluating matrix, as shown in Tables 1–4.

Actual cases: This stands for the number of attributes predicted by the model to be positive and the real is also positive; TP stands for actual case, which means the number of attributes predicted by the model to be positive and real is also positive; fake positives: The number of attributes the model predicts to be both positive and negative. False negatives: This is the number of attributes the model predicts to be both positive and negative. FP stands for “false positives” [22].

The proposed blockchain-based B-TLBO methods acquire a maximum 89.64% accuracy over the ODUM data set, whereas other methods acquire a maximum 79.52% accuracy, i.e., gain by SPTLBO as shown in Figure 4.

The proposed blockchain based B-TLBO methods acquire a maximum 79.52% *F*1-score over the ODUM dataset, whereas other methods acquire a maximum 69.65% *F*1-score, i.e., gain by SPTLBO as shown in Figure 5.

The proposed blockchain-based B-TLBO methods acquire a maximum 78.52% recall over the ODUM dataset, whereas other methods acquire a maximum 66.12% recall, i.e., gain by SPTLBO as shown in Figure 6. The proposed blockchain-based TLBO methods acquire a maximum 76.52% precision over the ODUM dataset, whereas other methods acquire a maximum 66.45% precision, i.e., gain by SPTLBO as shown in Figure 7.

## 5. Conclusion

In the teaching stage, the “expectation effect” theory in social psychology is introduced to simulate the phenomenon that teachers have higher expectations for outstanding students such that individuals with better fitness values can move closer to the optimal individual faster; in the learning stage, the theory of field dependence simulates the differences in the way students with different personalities acquire knowledge, to preserve the diversity of results better and avoid falling into local optimum; after the learning stage, a self-learning method adjustment stage is added to allow individuals to self-rank by adopting different strategies for learning, thereby effectively improving the optimization accuracy and convergence speed of the algorithm. This research paper, focusing on the defects of low optimization precision and slow convergence speed when solving complex optimization problems of the teaching and learning optimization algorithm, from the perspective of social psychology, combined with the changes of people's psychological emotions, improved the original teaching and learning optimization algorithm. To verify the algorithm's performance, 25 test functions are selected for numerical experiments. The results show that, compared with the original B-TLBO, PSO, GA, and IA algorithms, the SPTLBO algorithm proposed in this paper has fast convergence speed, high optimization accuracy, and stronger algorithm stability when solving low-dimensional and high-dimensional functions. This research looks at social psychology, bearing in mind human emotions and behaviors, and simulating the impact of human psychological factors on educational outcomes. It can be observed that taking human psychological elements into account while creating algorithms has a positive impact on algorithm performance. The target of TLBOs is to generate high-accuracy solutions as rapidly as feasible in recognized domains. This theory can be used to improve the teaching and learning algorithms in the early stages of learning, as well as to tackle more sophisticated optimization problems like dynamic vehicle path optimization, parameter optimization in numerous disciplines, and so on.

## Figures and Tables

**Figure 1:** Mental state relation to student.

**Figure 2:** Teacher learning phenomena.

**Figure 3:** Students' diversity.

**Figure 4:** Accuracy of physiological prediction.

**Figure 5:** *F*1-score of physiological prediction.

**Figure 6:** Recall of physiological prediction.

**Figure 7:** Precision of physiological prediction.

**Table 1:** Accuracy of physiological prediction.

Methods	Dataset			
	ICPSR	SAMHDA	NACJD	ODUM
SPTLBO	75.56	77.26	78.52	79.52
B-TLBO	81.56	85.05	86.35	89.64
PSO	79.52	76.52	74.23	76.25
GA	71.25	74.52	75.24	77.25

**Table 2:** *F*1-Score of physiological prediction.

Methods	Dataset			
	ICPSR	SAMHDA	NACJD	ODUM
SPTLBO	65.23	63.45	68.45	69.65
B-TLBO	74.52	81.56	78.56	79.52
PSO	64.52	66.85	69.45	70.56
GA	61.56	66.45	65.45	68.52

**Table 3:** Recall of physiological prediction.

Methods	Dataset			
	ICPSR	SAMHDA	NACJD	ODUM
SPTLBO	66.45	64.23	67.52	66.12
B-TLBO	75.62	80.23	79.52	78.52
PSO	61.25	64.25	67.52	69.23
GA	60.23	61.35	65.23	59.52

**Table 4:** Precision of physiological prediction.

Methods	Dataset			
	ICPSR	SAMHDA	NACJD	ODUM
SPTLBO	59.52	60.23	64.56	66.45
B-TLBO	70.23	75.56	77.52	76.52
PSO	60.41	62.23	67.45	64.12
GA	56.23	56.23	60.49	61.85

## Data Availability

The data shall be made available on request.

## References

[1] Alvi S. T., Uddin M. N., Islam L., Ahamed S. From conventional voting to blockchain voting: categorization of different voting mechanisms.

[2] Charla G.-B., Karen J., Miller H., Chun M. The Human-side of Emerging Technologies and Cyber Risk: a case analysis of blockchain across different verticals.

[3] Wong L.-W., Tan G. W.-H., Lee V.-H., Ooi K.-B., Sohal A. (2022). Psychological and system-related barriers to adopting blockchain for operations management: an artificial neural network approach. *IEEE Transactions on Engineering Management*.

[4] Xin K., Zhang S., Wu X., Cai W. Reciprocal crowdsourcing: building cooperative game worlds on blockchain.

[5] Kano Y., Nakajima T. An alternative approach to blockchain mining work for making blockchain technologies fit to ubiquitous and mobile computing environments.

[6] Zhao X. Teaching-learning based optimization with crossover operation.

[7] Zhao X. Improved teaching-learning based optimization for global optimization problems.

[8] Maity D., Ghosal S., Banerjee S., Chanda C. K. Bare bones teaching learning based optimization for combined economic emission load dispatch problem.

[9] Tuo S. Modified teaching-learning-based optimization algorithm.

[10] Ouyang H., Wang Q., Kong X. Modified teaching-learning based optimization for 0–1 knapsack optimization problems.

[11] Yao Q., Shabaz M., Lohani T. K., Wasim Bhatt M., Panesar G. S., Singh R. K. (2021). 3D modelling and visualization for vision-based vibration signal processing and measurement. *Journal of Intelligent Systems*.

[12] Raj A., Venkaiah C. Optimal PMU placement by teaching-learning based optimization algorithm.

[13] Crawford B., Soto R., Leiva F. A., Johnson F., Paredes F. The set covering problem solved by the binary teaching-learning-based optimization algorithm.

[14] Dhandhia A., Pandya V. Binary classification of static security assessment using teaching learning based optimization enhanced support vector machine.

[15] Godara J., Batra I., Aron R., Shabaz M., Lin H. (2021). Ensemble classification approach for sarcasm detection. *Behavioural Neurology*.

[16] Chen C.-H. Group leader dominated teaching-learning based optimization.

[17] Tiwari A., Dhiman V., Iesa M. A. M., Alsarhan H., Mehbodniya A., Shabaz M., Lin H. (2021). Patient behavioral analysis with smart healthcare and IoT. *Behavioural Neurology*.

[18] Chaudhary V., Yadav R., Panwar R. Design and analysis of a 5G electromagnetic shielding structure using teaching learning based optimization.

[19] Gupta A., Awasthi L. K. Peer enterprises: possibilities, challenges and some ideas towards their realization.

[20] Kwan H. K., Zhang M. Minimax design of linear phase FIR Hilbert transformer using teaching-learning-based optimization.

[21] Sharma C., Bagga A., Sobti R., Shabaz M., Amin R., Koundal D. (2021). A robust image encrypted watermarking technique for neurodegenerative disorder diagnosis and its applications. *Computational and Mathematical Methods in Medicine*.

[22] Qureshi S. R., Gupta A. Towards efficient big data and data analytics: a review.

